# Quantitative Evaluation of Small Intestinal Hemorrhage Using Energy Spectrum CT Iodine-Water Map

**DOI:** 10.1155/2022/9234579

**Published:** 2022-04-28

**Authors:** Lijuan Wen, Mingfei Zuo, Tian Bai, Xuejia Sun, Na Zhang, Jingqi Sun, Cuicui Wu, Li Wang

**Affiliations:** Radiographic Imaging Center, The Third Affiliated Hospital of Qiqihar Medical University, Qiqihar, 161000 Heilongjiang, China

## Abstract

The objective of this research is to analyze the quantitative evaluation of human small intestinal bleeding by observing and analyzing animal experiments of small intestinal hemorrhage in rabbit models for the convenience of understanding the role of energy spectrum CT iodine-water diagram in animal experimental research of quantitative evaluation of small intestinal bleeding in rabbit models. Compared with the energy spectrum of iodine-water graph of a rabbit CT model, the present study studied the quantitative evaluation of small intestinal bleeding by using a rabbit model instead of human. According to the method mentioned above and the analysis of experimental data, the role of energy spectrum CT iodine-water map and the quantitative evaluation of human small intestinal bleeding have been understood. It was found that the energy spectrum CT iodine-water map replaces humans in the rabbit model for quantitative evaluation of small intestinal bleeding in animal experiments, which is important in the present study. Besides, based upon the combination of theoretical and experimental data, the ten flow rates set on the base material iodine (water) maps of the arterial phase and the portal phase can be analyzed to detect the leakage of contrast agent. The yield was 100%. The research results showed that the animal experiment of quantitative assessment of small intestinal bleeding by replacing the human body with the rabbit model in the energy spectrum CT iodine-water diagram is critical to humans in the study of small intestinal hemorrhagic diseases. In addition, it can be used to adjust the treatment plan timely according to the amount of bleeding to prevent shock or heavy bleeding that threatens patients' lives.

## 1. Introduction

A traditional CT tube produced a continuous X-ray energy distribution. To be specific, the X-ray energy was mixed, and the obtained CT image showed an average effect of mixed energy, thus resulting in inaccurate CT values of the substance. It can be seen that fully demonstrating inherent characteristics is difficult [1]. Single-energy imaging of lesions of energy spectrum data and its special energy spectrum analysis tool can be easily obtained in energy spectrum CT which can directly show the change trend of CT values in the shape and position of energy spectrum curves of lesions between 40 and 140 keV [2]. Two different substances are used to express a specific density of tissue by means of material separation techniques. Water and iodine are common basic substances in spectral CT imaging. More importantly, iodine (water) density value can accurately reflect the enhancement degree of the lesion, provide a parameter more sensitive than the CT value, and accurately reflect the situation of the contrast agent entering the lesion [3].

After the application of energy spectrum CT in clinic, its various imaging technologies have achieved good results in the diagnosis of various system diseases of the human body. For example, at present, commonly used iodide maps can detect pulmonary embolism and assess pulmonary blood flow perfusion simultaneously; the basal material map can be used to analyze the content of basal material in the lesion for the sake of further lesion evaluation and analysis; the best single-energy image can show the lesion more clearly; on the other hand, the energy spectrum curve can be used to better analyze the different chemical components of the lesion. In addition, the spectrum CT can remove scleral artifacts, improve image quality, and better observe lesions [4].

Energy spectrum CT imaging may display varied X-ray energy absorption of different human tissues and morbid components and produce more comprehensive anatomical imaging of human tissues and organs, thus more clearly exhibiting the normal human body as well as diseased tissue. Furthermore, gem spectrum imaging technology may be utilized to evaluate the material properties of the human body and quantitatively assess the material composition. Furthermore, energy spectroscopy is the physical underpinning of energy spectroscopic imaging. Because X-rays are a kind of light, energy spectroscopy of X-rays may also be used to evaluate human body components. Small intestinal hemorrhage is clinically uncommon, manifesting as anemia, blood in the stool, or black stool, and accounts for 3.0 5.0 percent of total gastrointestinal bleeding. Because of the low incidence, clinical symptoms were hidden and there was a lack of specificity. Furthermore, the small intestine has long possessed intestinal length, a short mesentery, a folded abdominal cavity, and a significant activity. It is difficult to completely investigate traditional gastroscopy and colonoscopy. Nonetheless, it is important noting that there are always blind spots in practical therapy, and missed diagnosis, misdiagnosis, and misuse are common [5].

Experimental researches are taken as a tool in the present study to grasp the role of energy spectrum CT iodine-water diagrams and the quantitative evaluation of human small intestinal bleeding, as well as comparative exploration before and after application. Upon theoretical analysis and experimental exploration, energy spectrum CT iodine-water diagrams were found. The role of the rabbit model in the human experimental study of the quantitative evaluation of small intestinal bleeding is analyzed, processing the data through data recording, sorting, calculation, mapping, and analysis and using the energy spectrum CT iodine-water diagram to replace the human model with the small intestine. Plus, the quantitative evaluation of bleeding was performed on the statistical dataset of simulated animal experiments. Combined with the data, the function of iodine-water graph of the CT energy spectrum was analyzed empirically. Also, combined with the available data, the quantitative evaluation of human intestinal bleeding was summarized and analyzed. The results showed that with the method of the present study, the recognition rate reaches 46%.

## 2. Proposed Method

### 2.1. Energy Spectrum CT

Small intestine CT imaging (CTE) is a means to display the small intestine and large intestine using multislice spiral CT before taking a large amount of neutral contrast agent. Previous researches and practice have shown that CTE can clearly show the thickening of the intestinal wall, pelvic ileal ring, mesenteric fat, and mesenteric structure when compared with conventional small bowel follow-up examinations. Compared with capsule endoscopy and magnetic resonance examination, CTE can better evaluate the small intestine. It has been reported that small intestinal CTE has higher diagnostic accuracy for Crohn's disease. Full expansion of the small intestine is a prerequisite for the success of CTE. However, with the expansion of the intestine and the thinning of the intestinal wall, the degree of enhancement will also be weakened accordingly, thereby reducing the contrast of the fluid in the cavity. GSI technology can obtain 40140 keV single-energy image. According to the light point effect and the *K*-edge effect, the energy of the material is different. Under different energies, the material absorbs X-rays to different degrees, thus showing different densities and contrasts to obtain the best single-energy image. In order to improve image quality, MRC is an examination method in which the bowel is marked by oral or rectal infusion of gas, water, or paramagnetic or superparamagnetic iron oxide particle suspensions and intravenous injection of gadolinium contrast agent. Apparently, it has a high sensitivity for the diagnosis of colorectal cancer. MR-DWI features high accuracy in excluding lymph node metastasis, but it is easily affected by the cross section of small vessels in the abdomen and has a certain false-positive rate. Nonetheless, it is difficult to be widely used in clinical practice due to its small scanning range, long time, high cost, and numerous contraindications. [6].

As an imaging method combining functional imaging and morphological imaging, PET/CT reflects not only changes in anatomy but also the level of cellular metabolism [7]. Compared with traditional imaging methods, PET/CT has its own advantages in the imaging diagnosis and preoperative staging of colorectal cancer. PET-CT, as the main focus of colorectal cancer, has high 18F-FDG uptake, which can detect colorectal cancer very early. MDCT scan is the most commonly used examination technique in clinic because of the fast scan speed and high image quality of MDCT and the multiphase enhancement being able to provide an image of the entire abdomen. The detection rate and diagnostic accuracy of the tumor were improved according to the morphological characteristics and enhancement characteristics of the tumor. Energy spectral CT is based on traditional CT, from traditional single-parameter imaging to multiparameter imaging of energy spectral CT and from original mixed-energy imaging to multienergy energy spectrum imaging. By means of unique methods such as energy spectrum analysis, water iodine matrix, and single-energy imaging, the tumor stage and differentiation can be accurately evaluated in addition to further clarifying the diagnosis [8–10].

### 2.2. Small Bowel Bleeding

Gastrointestinal and colorectal diseases are more frequent than gastrointestinal bleeding. The small intestine accounts for 75% of the total length of the digestive tract [11]. The anatomy includes the duodenum, jejunum, and ileum. Narrow intestinal bleeding refers to jejunal and ileal bleeding under the Treitz ligament. Given that duodenal bleeding is more common and can be directly examined by gastroscopy, it does not belong to the scope of intestinal bleeding. It was found that some cases were repeatedly examined with gastroscopy and/or colonoscopy as it is not uncommon to miss diagnosis of gastroscopy and colonoscopy, with the continuous innovation and improvement of examination technology. Finally, the bleeding lesions were found under the microscope. An increasing number of scholars tend to replace the previously unknown OGIB with more specific intestinal bleeding. With the invention and application of capsule endoscope (CE) and double-balloon enteroscopy (DBE), the diagnosis rate of small intestinal bleeding has been increasing. However, its clinical application still has many limitations.

As the final diagnosis and treatment of small intestinal bleeding, surgery is mainly to remove the corresponding intestinal segment, including lesions (mainly wedge resection, bowel segment resection, and bowel segment resection + lymph node dissection). The extent of the resection depends on the extent and nature of the lesion. To be specific, the wedge-shaped small intestinal wall resection is feasible in terms of small intestinal bleeding caused by small hemangiomas and diverticulum; for vascular malformations, localized inflammatory diseases, small intestinal benign tumors, large hemangioma, and small intestinal bleeding caused by diverticulum, the corresponding segment can be removed. For small intestinal bleeding caused by malignant tumors of the small intestine, it is necessary to strive for radical surgery, including radical resection of the diseased intestinal segment (proximal and distal 10-20 cm intestinal segment and tumor mesenteric resection) and regional lymph node dissection. For patients who cannot undergo radical surgery, tumor burden can be minimized by means of palliative surgery on the basis of controlling intestinal bleeding. However, after all, surgical treatment is invasive. Plus, it is still considered as the ultimate method for the diagnosis and treatment of small bowel bleeding. Strict clinical indications include small bowel hemorrhage that cannot be qualitatively and locally diagnosed through clinical examinations such as imaging and endoscopy; small intestinal bleeding caused by vascular malformation that cannot be treated with intervention or is not effective; and local intestinal bleeding caused by local lesions or inflammatory bowel disease combined with intestinal obstruction, intestinal perforation, and massive hemorrhage. Small intestinal bleeding failed to respond to conservative treatment. Surgical treatment mainly includes traditional open surgery and laparoscopic surgery. Traditional open surgery features large surgical injury, long abdominal incision, and slow postoperative recovery.

In recent years, with the continuous improvement of laparoscopic surgery equipment, the continuous development of minimally invasive technology, and the accumulation of experience in the diagnosis and treatment of diseases in small bowel bleeding, laparoscopic surgery can also achieve the same effect as open surgery and has surgical trauma, small incision, rapid postoperative recovery, and low incidence of complications. The causes of small intestinal bleeding are mainly vascular diseases, tumors, inflammatory lesions, and small intestinal diverticulum. Vasculature is the main cause of small bowel disease, accounting for 70.0%-80.0%, followed by small bowel tumors, accounting for 5.0-10.0%. The main cause of small intestinal bleeding in China is small intestinal tumors, accounting for about 14.0%-40.0%, followed by vascular diseases or small intestinal diverticulum. The cause of small bowel bleeding varies by age. The main cause of small bowel bleeding in children is intussusception and Merkel diverticulum. With respect to adults under 50, small bowel tumors are the most common, followed by diverticulum, polyps, and Crohn's disease. In middle-aged and older patients over 60 years of age, the main cause of small intestinal bleeding is vascular disease, in addition to congenital vascular abnormalities. Reasons leading to such impacts include intermittent venous blood flow obstruction due to contraction into the gastrointestinal mucosa and slow venous blood flow caused by submucosal veins and circuitous expansion. Over a long period of time, it leads to the dilatation of mucosal capillaries and submucosal blood vessels, forming small bowel vascular lesions. Small bowel tumors are relatively rare in gastrointestinal tumors, accounting for about 2.0%. The most common site of small bowel tumors is the ileum, followed by the duodenum. The most common type of histopathology is carcinoid, followed by adenocarcinoma and lymphoma. Also, benign tumors are also more common, including leiomyoma, adenoma, and stromal tumor. The most common site of small bowel tumors is the duodenum, followed by the jejunum and ileum. The most common histopathological type is adenocarcinoma, followed by stromal tumors; benign tumors are stromal tumors; malignant tumors are adenocarcinomas; and malignant tumors are next. The peak age of Crohn's disease is 21-30 years. But it also takes place at 60-80 years. The overall proportion of women is slightly higher than that of men [12].

The application of conservative treatments such as hemostatic drugs and somatostatin and its derivatives will also reduce the positive diagnosis rate of small bowel vascular disease, which may be related to regional, ethnic, and genetic differences. The etiology of small intestinal bleeding in varying age groups is different. Besides, clinically rare causes include intestinal intussusception, intestinal torsion, hookworm disease, polyps, allergic purpura, systemic bleeding, radiation enteritis, and non-said drug factors, which may need different degrees of small intestinal bleeding. In addition, clinical attention is required as its clinical manifestations lack specificity and it is difficult to diagnose. Given that the small intestine is 5-6 meters long, the intestines overlap each other, and the activity is large. Barium meal in the digestive tract does not easily show the lesion. It is difficult to observe the small intestine with conventional endoscopy. Angiography and nuclide scans may also be restricted if small or slow interstitial bleeding took place in the small intestine. In the clinic, patients' lives are often threatened by repeated, persistent, or massive bleeding. Therefore, it should be diagnosed early and treated promptly. Although there are many examination methods for small intestinal bleeding, the diagnosis of small intestinal bleeding is still a difficult problem due to the lack of specificity of clinical manifestations, the particularity of small intestine anatomy, and the limitations of various examination methods. Screening can be performed through gastroscopy and colonoscopy, and then, abdominal CT was enhanced. Plus, CTA and CT colonoscopy can be improved when necessary. For repeated small amounts of gastrointestinal bleeding, capsule endoscopy or enteroscopy can be improved; with respect to patients with gastrointestinal bleeding, DSA or ECT can be used, or superselective arterial embolization can be used. After all, the laparoscopy has a very good application value in the diagnosis and treatment of small intestinal bleeding. With the advancement of science and technology, more and more examination methods have been applied to the diagnosis and treatment of small bowel bleeding, while each has its advantages and disadvantages, mainly including enteroscopy: the scope that can be controlled by enteroscopy observation for realizing direct observation of the small intestine can be divided into oral and anal examination methods. Not only the mucosal surface of the small intestine can be directly observed, but also the location of the small intestinal bleeding and the cause of the small intestinal bleeding can be found. It can also be used for endoscopic biopsy and treatment.

### 2.3. Quantitative Evaluation

Material separation and quantitative measurement are one of the important functions of EDCT. According to the law of expression of undetermined substances in X-ray absorption, the materials were separated by matrix-pair ratio after CT scan of gemstone spectrum, and the separated base materials could be used for quantitative analysis. This method breaks through the defect that traditional CT only relies on CT for analysis. In this case, unmeasured substances can be displayed clearly and quantitatively. Besides, the changes of tissues, organs, and pathological changes can be clearly found via the quantitative analysis of the substance. This is conducive to the qualitative analysis of pathological changes and the judgment of pathological changes.

With the emergence of multislice spiral CT, the CT inspection technology has been constantly reformed and improved, and the number of detectors has rapidly developed from a simple single row to 2, 4, 16, 64, 256, 320, and so on. New imaging technologies and image postprocessing technologies have been mushroomed, and their clinical application value continues to increase. In recent years, dual-spectrum CT has achieved a transition from traditional mixed-energy to single-energy imaging, which has become a new climax in clinical and imaging research. Dual-energy CT imaging is the core technology to achieve high-low dual-energy (80 kV and 140 kV) switching. Its detector is a gemstone, which is able to generate dual-energy data and analyze the change of attenuation values of different materials with energy. When combined with the GSI software platform, it can provide conventional material separation and quantitative analysis, material density image, single-energy image, comprehensive analysis of energy spectrum, and other functions and provide more information for clinicians to diagnose diseases. And relevant outcomes have been achieved in practice. At present, spectral CT has made significant progress in the removal of scleral artifacts, kidney stones, pulmonary embolism, and tumors. At present, there are three main types of dual-energy CT: one is GE's single-source dual-energy CT, which is equipped with a set of bulbs and a set of detectors and quickly switches to 80/140 kV (usually <0.5 ms) through a single tube, which can collect two sets of energy data in real time; the other is Siemens dual-source dual-energy CT equipped with dual tubes and dual detectors. In addition, these two sets of tubes and detectors have been arranged vertically in the same frame, thus allowing two sets of energy collected data at the same time and in the same direction; the other is a dual-source single-source dual-energy CT equipped with a set of tubes and two sets of detectors. At present, however, this single-source dual-energy CT has not been used in clinical practice.

### 2.4. Energy Spectrum CT Image Reconstruction

#### 2.4.1. Traditional X-CT Imaging

X-CT imaging is the result of the interaction between X-rays and objects. In the presence of photoelectric effect, Compton scattering and electron pair take effects when X-rays pass through the object under test, some of the rays are absorbed, and the intensity of the rays will be attenuated. *μ* represents the linear attenuation coefficient of the measured object. When the X-ray with total incident photon number *I*_0_ passes through a uniform measured object with a thickness of 1, its attenuation law obeys the Lambert-Beer law, and the number of photons after passing through the object *I* is

(1) $$\begin{array}{c} I=I_{0}e^{-\mu l}. \end{array}$$

In the actual situation, the density distribution of the measured object is nonuniform. At this time, the measured object needs to be divided into n uniform units in the X-ray scanning direction. *μ*_1_, *μ*_2_, ⋯, *μ*_*n*_ represents the attenuation coefficient of each unit, and *l*_1_, *l*_2_, ⋯, *l*_*n*_ represents the corresponding length. Then, there is

(2) $$\begin{array}{c} I=I_{0}e^{-\left(\mu_{1}l_{1}+\mu_{2}l_{2}+\cdots +\mu_{n}l_{n}\right)}=I_{0}e^{-\sum \mu_{i}l_{i}}. \end{array}$$

When *n* tends to infinity, formula (2) becomes

(3) $$\begin{array}{c} I=I_{0}e^{-\int_{l}\mu \left(l\right)dl}. \end{array}$$

∫_*l*_*μ*(*l*)*dl* is the line integral of the attenuation coefficient of the measured object on the X-ray path 1, and its value is equal to the natural logarithm of the ratio of the number of photons before passing through the measured object and the number of photons that are not attenuated after passing through the measured object. In other words, the projection measurement value *p* is

(4) $$\begin{array}{c} p=\int_{l}\mu \left(l\right)dl=\ln\left(\frac{I_{0}}{I}\right). \end{array}$$

CT image reconstruction is the process of estimating the object attenuation coefficient *μ* through the projection data *p*.

#### 2.4.2. Energy Spectrum CT Imaging Principle

The traditional X-CT energy integration detector was replaced with a photon counting detector. By setting a reasonable energy threshold, the number of photons was calculated by the energy channel when the incident photon passes through the object to be measured. And the collected attenuated photon information was used to obtain the multienergy spectrum imaging of the measured object which is based on the energy spectrum CT imaging principle of the photon counting detector.

Assume the incident photon intensity of the X-ray continuous energy spectrum is *I*_0_. According to the Lambert-Beer law and the energy threshold which is set to *T*_1_, the photon intensity received by the photon counting detector is

(5) $$\begin{array}{c} I\left(T_{1}\right)=\int_{T_{1}}^{\infty }I_{0}\left(E\right)D\left(E\right)\exp\left(-\int_{L}\mu \left(E,l\right)dl\right)dE, \end{array}$$

wherein *D*(*E*) is the detector efficiency. *μ*(*E*, *l*) represents the linear attenuation coefficient on the *l*th path under energy *E*.

The photon intensity received by the photon counting detector is

(6) $$\begin{array}{c} I\left(T_{1},T_{2}\right)=\int_{T_{1}}^{T_{2}}I_{0}\left(E\right)D\left(E\right)\exp\left(-\int_{L}\mu \left(E,l\right)dl\right)dE. \end{array}$$

Similar to traditional X-CT, let us take the logarithm of formula (6) to get the projection value in the given energy segment *E*(*T*_1_, *T*_2_):

(7) $$\begin{array}{c} P=\ln\left(\frac{\int_{T_{1}}^{T_{2}}I_{0}\left(E\right)D\left(E\right)dE}{\int_{T_{1}}^{T_{2}}I_{0}\left(E\right)D\left(E\right)\exp\left(-\int_{L}\mu \left(E,l\right)dl\right)dE}\right). \end{array}$$

#### 2.4.3. The Basis of CT Image Reconstruction

*(1) Radon Transformation and Inverse Transformation*. Given a function, *f*(*x*_1_, *x*_2_), the Radon transformation refers to the line integral of the function *f*(*x*_1_, *x*_2_) along the line *z* given by the plane, where *φ* and *u* are the position parameters of the line *z*; then, the Radon transformation and its inverse transformation are expressed as

(8) $$\begin{array}{c} p=\int_{-\infty }^{\infty }f\left(x_{1},x_{2}\right)dz=\int_{-\infty }^{\infty }\hat{f}\left(r,\theta \right)dz=\int_{-\infty }^{\infty }\hat{f}\left(\sqrt{u^{2}+z^{2}},\varphi +{tg}^{-1}\frac{z}{u}\right)dz,\\ \hat{f}\left(r,\theta \right)=\frac{1}{2\pi^{2}}\int_{0}^{\pi }\int_{-\infty }^{\infty }\frac{1}{r\cos\left(\theta -\varphi \right)-u}\frac{\partial p}{\partial u}dud\varphi . \end{array}$$

#### 2.4.4. Fourier Central Slice Theorem

Fourier center slice theorem is the theoretical basis to use projection to reconstruct images. Assume that under the viewing angle *θ*, the projection data of the tomographic image *f* (*x*, *y*) of the measured object is *g* (*t*, *θ*), and its one-dimensional Fourier transform*G* (*w*, *θ*)is equivalent to the image*f* (*x*, *y*). The two-dimensional Fourier transform has a slice of*F*(*ω*_1_, *ω*_2_), and the slice passes through the origin of coordinates and intersects the*ω*_1_axis at an angle of*θ*degrees. Select the rotating coordinate system *ts* at the origin of the *xy* plane coordinate system; then, set the coordinate axis *s* to be parallel to the incident X-ray photon beam, and set the coordinate axis *t* perpendicular to the incident X-ray photon beam. In the *xy* plane coordinate system, *f* (*x*, *y*) can be represented by *f*′(*t*, *s*) of the *ts* rotating coordinate system, and the *xy* plane coordinate system and the *ts* rotating coordinate system satisfy the following formulas:

(9) $$\begin{array}{c} t=x\cos\theta +y\sin\theta \\ s=-x\sin\theta +y\cos\theta . \end{array}$$

Let *g* (*t*, *θ*) be the line integral along the straight line *s*, which is the projection of the rotating coordinate system *t*-*s* under the viewing angle *θ*; then, the formula is

(10) $$\begin{array}{c} g\left(t,\theta \right)=\int_{-\infty }^{+\infty }f^{\prime }\left(t,s\right)ds. \end{array}$$

Let*t*be a variable, one-dimensional Fourier transform which is performed on the projection*g* (*t*, *θ*)to obtain

(11) $$\begin{array}{c} G\left(\omega ,\theta \right)=\int_{-\infty }^{+\infty }g\left(t,\theta \right)e^{-j2\pi \omega t}dt=\int_{-\infty }^{+\infty }\int_{-\infty }^{+\infty }f\left(x,y\right)e^{-j2\pi \omega \left(x\cos\theta +y\sin\theta \right)}dxdy. \end{array}$$

And the two-dimensional Fourier transform *F*(*ω*_1_, *ω*_2_) of *f* (*x*, *y*) can be expressed as

(12) $$\begin{array}{c} F\left(\omega_{1},\omega_{2}\right)=\int_{-\infty }^{+\infty }\int_{-\infty }^{+\infty }f\left(x,y\right)e^{-j2\pi \omega \left(x\omega_{1}+y\omega_{2}\right)}dxdy. \end{array}$$

Let formula (11) be equal to formula (12); at this time, the following relationship is shown as below:

(13) $$\begin{array}{c} \omega_{1}=\omega \cos\theta ,\\ \omega_{2}=\omega \sin\theta . \end{array}$$

The expression of Fourier's central slice theorem is

(14) $$\begin{array}{c} G\left(\omega ,\theta \right)=F\left(\omega \cos\theta ,\omega \sin\theta \right). \end{array}$$

#### 2.4.5. Joint Algebraic Reconstruction Algorithm for Ordered Subsets (OS-SART)

Initialize the image *f* to be reconstructed, let *f*_0_ = 0, and divide the projection data *P* into *T* ordered subsets:

(15) $$\begin{array}{c} \underset{1\leq t\leq T}{\cup }S_{t}=\left\{1,2,\cdots ,I\right\},\\ t=k\mathrm{mod}\left(T\right)+1. \end{array}$$

Calculate the estimated value of the projection corresponding to a ray in a certain direction in the *t*^th^ subset:

(16) $$\begin{array}{c} {\hat{p}}_{i}=\overset{J}{\underset{j=1}{\sum }}a_{ij}f_{j}^{k},\;i\in S_{t}. \end{array}$$

Correct the reconstructed image by using the OS-SART algorithm; *k* is the number of iterations:

(17) $$\begin{array}{c} f^{k+1}=f^{k}+\lambda_{k}\cdot \underset{i\in S_{t}}{\sum }\frac{a_{ij}}{\sum_{i\in S_{t}}a_{ij}}\frac{p_{i}-{\hat{p}}_{i}}{\sum_{j=1}^{J}a_{ij}}. \end{array}$$

The problem of energy spectrum CT reconstruction can be expressed as

(18) $$\begin{array}{c} \min{\left\|{Af}_{E}-P_{E}\right\|}_{2}^{2}. \end{array}$$

The discrete gradient transform of image *f* is defined as

(19) $$\begin{array}{c} \nabla f_{ij}=\sqrt{{\left(f_{i+1,j}-f_{ij}\right)}^{2}+{\left(f_{i,j+1}-f_{ij}\right)}^{2}}. \end{array}$$

Its TV is defined as

(20) $$\begin{array}{c} \text{TV}\left(f\right)={\left\|\nabla_{\text{TV}}f\right\|}_{1}=\underset{i}{\sum }\underset{j}{\sum }\sqrt{{\left(f_{i+1,j}-f_{ij}\right)}^{2}+{\left(f_{i,j+1}-f_{ij}\right)}^{2}}. \end{array}$$

Therefore, the objective function of CT reconstruction based on TV minimization is

(21) $$\begin{array}{c} \underset{f}{\min}{\left\|{Af}_{E}-P_{E}\right\|}_{2}^{2}+\lambda \text{TV}\left(f_{E}\right). \end{array}$$

This section proposes the above method for experimental research; the specific process is shown in Table 1.

## 3. Experiments

### 3.1. Experimental Materials

CT scanner, micropump wzs-50f6 dual-channel micropump, and authoritative institutions regularly calibrate micropump indicators. The specifications of the venous indwelling needle are 24 g × 0.75 and 0.7 mm × 19 mm. The micropump extension tube is a common type. The contrast agent iohexol has a standard of 300 mgi/M1. Iod oxitol and normal saline were mixed in a volume ratio of 1 : 45 to simulate enhanced blood. First, add a rebel to a 50 ml syringe, fix the syringe on the micropump, adjust the micropump, and simulate the active small intestine with a flow rate of 0.1, 0.2, 0.4, 0.6, 0.8, 1.0, 1.2, 1.4, 1.6, and 1.8 ml/min bleeding. New Zealand white rabbit colon animal model was provided by the Animal Experiment Center of Henan Province. Six New Zealand white rabbits were fed under the same conditions. Before the experiment, the gastrointestinal tract of rabbits was fully dilated by gavage to simulate the intestinal preparation of the small intestine. In the experiment, the rabbits were killed and their internal organs were exposed.

### 3.2. Experimental Methods

In this experiment, the prepared contrast agent was pumped into a 60 ml syringe, fixed on a micropump, and connected to a micropump connection tube. Precontrast was added to the test tube. One end of a standard 24 G venous indwelling needle was connected to a micropump extension tube. The other end was connected to the colon of the white rabbit. Also, it is noteworthy that the needle must pass through the intestinal wall, fix the fixed needle on the intestinal wall, and then adjust the micropump. The injection flow rates were 0.1, 0.2, 0.4, 0.6, 0.8, 1.0, 1.2, 1.4, 1.6, and 1.8 ml/min. The scanning conditions are as follows: dual-energy GE discovery HD 75064 layer CT energy spectrum mode uses scanning; tube voltage was set to be 80/140 kV (0.5 ms) instantaneous switching. The tube current was set as 600 mA, screw spacing was set as 0.984, and X-ray tube speed was adjusted to 0.8 s/rot; the number of scan layers was set to be 16, and the layer thickness and layer interval were adjusted to 5.0 mm. After that, the reconstruction of the original image obtained was 1.25 mm in thickness and interval and then transferred to the ADW4.5 workstation for postprocessing. The scanning method is dual-energy GE discovery HD 75064 line CT. After injection of contrast agent, scans were delayed 15 s, arterial phase, and 40 s, and portal phase. Then, the blood flow rate of each group was scanned once during the arterial phase and the portal phase.

In this part, the above steps were proposed for the experiment of animal experimental study on quantitative evaluation of small intellectual hemorrhage with a rabbit model instead of the human body using energy spectrum iodine-water map.

## 4. Image Analysis

The seven single-energy images of 40 keV, 50 keV, 60 keV, 70 keV, 80 keV, 90 keV, and 100 keV were obtained using standard reconstruction methods according to data obtained from dual-energy CT energy spectrum mode scanning. The corresponding iodine (water) base map was obtained after processing at the workstation. Then, a clear observation of a single 60 keV energy contrast agent in the secretory area and the image of the local ROI base material iodine (water) base was based on the selection of the base iodine (water). All the exudate contrast agents can be observed in the current. Plus, the layer must be included in the area of interest of the measurement. GSI tends to scan under the conditions, through which we could measure the iodine concentration of the contrast agent exudate layer and the portal phase for the convenience to observe the contrast agent iodine concentration of the exudate layer as well as the measured area of the contrast agent secretion area in the arterial phase and the portal vein. Moreover, in the measurement phase of the portal vein, the background can be observed with the content of iodine in the small intestine and the mean *ρ*. The background can be taken (the area of the portal vein is the same stage) to calculate the sum of the iodine content inexudation zone of the contrast medium in the portal phase and the sum of the iodine content in the background of the volume difference in the exudation zone of the two contrast agents. Finally, the difference in iodine content between the portal and arterial calculation stages, *Δ*IC (*Δ*IC = IC arterial phase integrated circuit IC portal segment background), is calculated. The blood flow calculation formula is *v* = ΔIC/(Δ*t* × *ρI*). The unit of*v*measurement is milliliters per minute;Δ*t* = 25 s, scanning interval portal segment, and arterial phase; and*ρ*concentration of iodized contrast injection, in micrograms per cubic centimeter. Before the commencement of this experiment, under the same scanning conditions as described above, we can fill a 50 ml syringe to prepare the contrast agent, scan with GSI mode, select the basic map of iodine (water) corresponding to the observation of a single-energy 60 keV, select a relatively uniform five layers of iodine contrast agent (water) basic image, measure the iodine concentration (the same area) of these five layers, and take the average value (*ρ*). At this point, the flow of active small intestinal bleeding without bowel preparation can be calculated and the amount of small intestinal bleeding can be assessed. In case of objections to measurements, discussing and resolving them would be favored solutions. The 10 flow rates were measured 5 times, respectively, and then averaged. In the calculation method, if you can see 10 layers of contrast agent scanned in the first stage, then in each layer, the iodine content (IC) = iodine concentration ROI (100ug/cm^3^) × ROI region layer thickness (Mm), the area and iodine concentration can be directly from the iodine (water) base map, and the thickness of the scan layer is 1.25 mm; the analysis was performed using SPSS17.0 statistical software, and the paired *t* test was taken to analyze the measured bleeding volume and the actual bleeding volume. The result showed that the difference was statistically significant (*P* < 0.05); the relationship between the measured value and the actual value of the bleeding volume was obtained by linear regression analysis, and the regression equation was obtained.

## 5. Discussion

### 5.1. Analysis of Detected Contrast Agent

#### 5.1.1. Analysis of Detection Rate

According to the statistical analysis of the data shown in Figure 1 and Table 1, when the true flow rate was 1.8 ml/min, 31 layers of contrast medium exudation were detected in the arterial phase, and 40 layers of contrast medium exudation were detected in the portal phase. At a flow rate of 1.6 ml/min, 16 layers of contrast medium exudation were detected in the arterial phase and 28 layers of contrast medium exudation were detected in the portal phase; when the true flow rate was 1.4 ml/min, 11 layers of contrast agent were secreted in the artery phase detection; when the flow rate is 1.0 ml/min, the number of layers of contrast agent exudate was 16, 23, and 0.8 ml/min; when the flow rate was 0.6 ml/min, the flow rate on the 17th, the flow rate is 22; when the flow rate was 0.4 ml and when the flow rate was 10/min, the flow rate was 29; when the true flow rate was 0.2 ml/min, the number of layers detected in the arterial phase was 14 layers, and the number of layers detected in the portal phase was 15 layers; when the true flow rate was at 0.1 ml/min, 7 layers were detected in the arterial phase and 9 layers were detected in the portal phase. The exudation of the contrast agent could be detected by setting 10 flow rates on the arterial and portal phase substrate iodine (water) maps, and the detection rate was 100%.

#### 5.1.2. Difference Analysis

According to the statistical analysis of the data shown in Figure 2 and Table 2, when the actual flow rate was 0.1 ml/min, the average value of the measured flow rate is 0.132 ml/min, and the error was 32.00%; when the actual flow rate was 0.2 ml/min, the average value of the measured flow was 0.230 ml/min, and the error was 15.00%; when the actual flow was 0.4 ml/min, the average of the measured flow was 0.456 ml/min, and the error was 14.00%; when the actual flow was 0.6 ml/min, when the average flow rate was 0.688 ml/min, the error was 14.67%; when the actual flow rate was 0.8 ml/min (Table 3), the average value of the measured flow rate was 0.928 ml/min, and the error was 16.00%; when the actual flow rate was 1.0 ml/min, the average value of the measured flow rate is 1.176 ml/min, and the error was 17.60%; when the actual flow rate was 1.2 ml/min, the average value of the measured flow rate was 1.400 ml/min, and the error was 16.67%; when the actual flow rate was at 1.4 ml/min, the average value of the measured flow was 1.6l4 ml/min, and the error is 15.29%; when the actual flow was 1.6 ml/min, the average of the measured flow is 1.846 m1/min, and the error was 15.38%; when the actual flow rate was 1.8 ml/min, the average value of the measured flow rate was 2.062 ml/min, and the error was 14.56% (Figure 3). When the measured flow rate was 0.2 ml/min (including 0.2 ml/min), the error gradually decreased, then stabilized as the actual flow rate increased. Then, it was in a lower state. The difference between the measured flow rate and the actual flow rate gradually decreases. Before the measurement flow rate was 0.2 ml/min, the error was large, indicating that the lower actual flow rate means greater effect on the contents of the intestinal tract.

### 5.2. Data Correlation Analysis

#### 5.2.1. Regression Analysis

According to the statistical analysis of the data given in Figure 1 and Table 1, when the real flow rate was 1.8 ml/min, 31 layers of contrast media exudation were discovered in the arterial phase and 40 layers were detected in the portal phase. When the flow rate was 1.6 ml/min, 16 layers of contrast medium exudation were detected in the arterial phase and 28 layers of contrast medium exudation were detected in the portal phase; when the true flow rate was 1.4 ml/min, 11 layers of contrast agent were secreted in the artery phase detection; when the flow rate was 1.0 ml/min, the number of layers of contrast agent exudate was 16, 23, and 0.8 ml/min; when the flow rate was 10/min, the flow rate was 29; when the true flow rate was 0.2 ml/min, 14 layers were detected in the arterial phase and 15 layers were detected in the portal phase; when the true flow rate was 0.1 ml/min, 7 layers were detected in the arterial phase and 9 layers were detected in the portal phase. The detection rate of contrast agent exudation was 100% when 10 flow rates were placed on the arterial and portal phase substrate iodine (water) maps.

#### 5.2.2. Error Rate Analysis

According to the statistical analysis of the data provided in Table 4 and Figure 4, the greatest inaccuracy is 32.00 percent when the correct flow rate is 0.1 ml/min. The smallest inaccuracy is 14.00 percent when the correct flow rate is 0.4 ml/min. The success percentage of colonoscopy varies according to study. Enteroscopy should be conducted after a modest amount of bleeding or no bleeding, since significant amounts of bleeding and high intestinal blood concentrations will impair judgment and observation of bleeding sites and lesions. However, enteroscopy is not widely used at the moment. The damaged intestinal wall and the exterior of the gut cannot be seen. At the same time, mastering enteroscopy is challenging. The procedure took a long time, and the patient was in a lot of discomfort. And with perforation, some patients cannot endure the difficulties, limiting the clinical use of colonoscopy to some degree (Figure 5). At the moment, digital subtraction selective arteriography (DSA) is the gold standard for gastrointestinal bleeding diagnosis. DSA should be evaluated initially in patients with gastrointestinal bleeding more than 0.5 ml/min. The more the bleeding, the higher the DSA positive rate, and the diagnostic accuracy rate may range from 12% to 69%. The majority of patients had angiography leakage and could be treated promptly with vascular embolization and medication therapy. The rate of hemostasis was high, particularly given the volume of bleeding. Tumors and vascular lesions, for example, are common causes of minor intestinal bleeding in patients. DSA had a greater incidence of active gastrointestinal bleeding diagnosis and a lower rate of active gastrointestinal bleeding diagnosis (Table 5).

### 5.3. Energy Spectrum CT Experimental Analysis

#### 5.3.1. Numerical Simulation Experiment

In the numerical simulation experiment, the equidistant fan beam scanning method was adopted. It showed that the scanning radius was 100 mm, the object radius was 12 mm, and the detector length was 40 mm. There were 320 detector units, and the size of each detector unit was 0.0625 mm. The voltage used in the simulation experiment was 120 kVp, and the energy spectrum distribution graph was generated by the SpectrumGUI software (Table 6). The simple model used in the simulation experiment consisted of 8 circular objects, including 5 materials.

1. PSNR represents the numerical indicators commonly used to measure image quality to verify the experimental results. The specific results are shown in Table 7 and Figure 6

By observing the data in the table, we can more intuitively find that the image reconstructed by the algorithm in the present study is closer to the real image provided by the experimental template. It further verifies the superior performance of the algorithm proposed in the present study in the data full sampling mode.

(2) The proposed algorithm has been verified in the present study by designing a simple model and a clinical rabbit model generated by MOBY software. In this way, the practicability of complex models and high-noise models can be obtained. Equidistant fan beam scanning mode was adopted, the scanning radius was 100 mm, the object radius was 10 mm, and the detector length was 20 mm. There were 320 detector units; each detector unit was 0.0625 mm in size. There were 360 angle projections collected uniformly in one scan data. The voltage used in the simulation experiment was 50 kVp, and the energy spectrum distribution diagram was generated by the SpectrumGUI software, as shown in Table 8 and Figure 7

In the present study, OS-SART iterative reconstruction is used to solve the fidelity term, and the number of subsets is selected as 5. In the a priori-based reconstruction algorithm, the reference image is reconstructed using the SB (Split Bregman) algorithm under the full spectrum channel of the simulation model.

## 6. Conclusions

1. Energy spectrum gem spectrum CT has been used to diagnose active gastrointestinal bleeding as it has been widely applied and further developed. Spectral CT iodine (water) substrate imaging has achieved certain outcomes in the qualitative and quantitative diagnosis of active intestinal bleeding
2. Using a single-energy image and iodine (water) image, we can make a qualitative diagnosis of active small intestinal bleeding without preparing the digestive tract and measure the flow of active small intestinal bleeding simultaneously. In this case, it is feasible to evaluate small intestinal bleeding active in nonideal conditions
3. It is believed that the value of energy spectrum CT in the quantitative diagnosis of active intestinal bleeding will be increasingly valued by imaging doctors and clinicians in the future. In addition, it can be widely used in clinical practice to better serve patients

## Figures and Tables

**Figure 1:** The experimental steps of the present study.

**Figure 2:** Detection rate analysis.

**Figure 3:** Difference analysis.

**Figure 4:** Regression analysis.

**Figure 5:** Error rate analysis.

**Figure 6:** Image quality metrics.

**Figure 7:** Energy spectrum of 50 kVp simulated voltages.

**Table 1:** Part of the technical flow chart of this method.

Proposed method	2.1	Energy spectrum CT
	2.2	Small bowel bleeding
	2.3	Quantitative evaluation
	2.4	Energy spectrum CT image reconstruction

**Table 2:** Detection rate analysis.

Classification	True flow rate (ml/min)									
	0.1	0.2	0.4	0.6	0.8	1	1.2	1.4	1.6	1.8
Arterial phase	7	14	10	17	15	16	20	11	16	31
Portal phase	9	15	29	22	24	23	30	26	28	40

**Table 3:** Difference analysis.

Injection rate	0.1	0.2	0.4	0.6	0.8	1	1.2	1.4	1.6	1.8
1	0.14	0.24	0.46	0.7	0.94	1.18	1.4	1.56	1.93	1.95
2	0.12	0.24	0.44	0.69	0.91	1.15	1.44	1.61	1.78	2.07
3	0.14	0.21	0.46	0.68	0.91	1.16	1.38	1.66	1.86	2.08
4	0.15	0.21	0.46	0.69	0.94	1.19	1.38	1.67	1.78	2.06
5	0.11	0.25	0.46	0.68	0.94	1.2	1.4	1.57	1.88	2.15
Average measured flow rate	0.132	0.23	0.456	0.688	0.928	1.176	1.4	1.614	1.846	2.062
Error rate	0.32	0.15	0.14	0.147	0.16	0.176	0.167	0.153	0.154	0.146

**Table 4:** Regression analysis.

*P* value	*r* value	*t* value	Scope of *P* value
0.00008	1	5.033	<0.001

**Table 5:** Error rate analysis.

True flow rate	Error rate
0.1	32.00%
0.2	15.00%
0.4	14.00%
0.6	14.70%
0.8	16.00%
1	17.60%
1.2	16.70%
1.4	15.30%
1.6	15.40%
1.8	14.60%

**Table 6:** Geometric parameters and composition of the model.

Object	Center coordinates (cm)	Long and short axis length (cm)	Material
1	(0.0001, 0.0001)	(0.8000, 0.8000)	Soft tissue
2	(0.0003, 0.0005)	(0.1200, 0.1200)	Air
3	(0.0041, 0.0056)	(0.1800, 0.1800)	Blood
4	(0.0074, 0.0079)	(0.1800, 0.1800)	0.3%gold + 99.7%blood
5	(0.0082, 0.0093)	(0.1800, 0.1800)	0.3%iodine + 99.7%blood

**Table 7:** Image quality metrics.

Algorithm	Ideal data for simulation		Simulated actual data	
	Blood	Water	Blood	Water
E-ART	36.7124	42.5362	31.1026	38.1765
ASD-NC-POCS	41.3567	49.1124	39.1534	47.1035
This article	54.0612	61.4632	51.2451	57.4106

**Table 8:** Energy spectrum of 50 kVp simulated voltages.

Energy (keV)	Photons/mm^2^ (keV)
10	1,129
20	4,231
30	15,672
40	11,236
50	873

## Data Availability

The datasets generated during and/or analyzed during the current study are available from the corresponding author on reasonable request.
